# Model of Human Tongue Squamous Cell Lines Stably Transfected with Human Papillomavirus (HPV)16 E6 and E7 Genes and Biological Characteristic Analysis

**DOI:** 10.1155/2021/9968691

**Published:** 2021-06-17

**Authors:** ZiLian Lan, Ziyao Jia, Hengyuan Guo, Zhaoshou Yang, Zifan Yang, Xuan Pan

**Affiliations:** ^1^Scientific Research Center of the First Affiliated Hospital of Guangdong Pharmaceutical University, Guangdong Pharmaceutical University, Guangzhou, Guangdong, China; ^2^Oral Research Center of the First Affiliated Hospital of Guangdong Pharmaceutical University, Guangdong Pharmaceutical University, Guangzhou, Guangdong, China; ^3^Examination Section of the First Affiliated Hospital of Guangdong Pharmaceutical University, Guangdong Pharmaceutical University, Guangzhou, Guangdong, China; ^4^Department of Biochemistry, Zhongshan School of Medicine, Sun Yat-sen University, Guangzhou, China

## Abstract

**Background:**

Human tongue squamous cell carcinoma (TSCC) is the most common oral cancer with the highest human papillomavirus (HPV) infection rate in oral cancer. The purpose of this study was to research the correlation between HPV and TSCC.

**Method:**

Plasmid pEGFP/HPV16 E6E7 and plasmid pEGFP/no HPV16 E6E7 were constructed. TSCC cell lines SCC9 and SCC15 were infected by liposome transfection and would be highly selected by antibiotic. Fluorescence imaging, PCR, and Western blot were used to detect the expression of HPV16 E6E7 in cells. The biological characteristics were detected by CCK-8, wound healing assay, qRT-PCR, and Western blot.

**Result:**

TSCC cell lines transfected with HPV16 E6E7 gene were successfully established and identified. And the proliferation and migration ability of the TSCC cell lines infected with HPV16 E6E7 gene were significantly stronger than that of the blank group.

**Conclusion:**

TSCC cell lines infected with HPV16 E6E7 with significantly higher ability of proliferation and migration were more malignant than those not infected with HPV16 E6E7.

## 1. Introduction

Oral cancer is the sixth most common cancer in the world, with high morbidity and mortality, accounting for more than 50% of confirmed patients, among which human tongue squamous cell carcinoma (TSCC) is the most common oral cancer [1]. Due to the poor accuracy of imaging detection, insufficient specificity of biomarkers, difficult clinical diagnosis, and the heavy burden of medical expenses in treatment options such as radiotherapy, chemotherapy, immunotherapy, and surgery, the survival and prognosis in oral squamous cell carcinoma (OSCC) are particularly poor, which cannot be significantly improved in the past century [2, 3].

In the 21st century, with oral sexual behavior appearing in the young people, human papillomavirus- (HPV-) associated oral cancer happens more and more frequently possibly due to the virus of sexual transmission [4, 5]. With the increasing number of cases of HPV-related oral cancer, the correlation between sexual behavior and oral cancer is becoming increasingly clear [6]. What is more, the ever-creasing clinical epidemiological and experimental evidence in recent decades also shows that oral cancer has close relationships with sexual behavior such as oral-vagina, oral-anal, and oral-penis [7–9]. But it is a comfortable and encouraging finding that HPV-associated OSCC have better clinical prognosis: the reported 3-year and 5-year OS rates even, respectively, increased to 93% and 89%, which means HPV has a promising effect on improving the prognosis of patients with oral squamous cell carcinomas [10, 11].

Although the mechanism of this encouraging effect has not been fully understood, the detection of biomarkers for the sensitivity and specificity of human OSCC associated with HPV has been compared and clarified, among which HPV16, E6, and E7 have been studied and discussed most frequently [12]. HPV16 plays a dominant role in HPV16, 18, 31, 45, 33, 52, 58, 35, 59, 56, 51, 6, 39, 68, 82, 66, 70, and 73 and infuses 46-63% squamous cell carcinoma, followed by HPV18 (10-14%) [13]. As for their positive roles in OSCC, multiple pathogenic factors and signaling pathways such as P16, P53, RB, E6, E7, and EGFR were studied in clinical cases and experimental observations [14]. However, whether and how HPV plays an effective regulatory role in changing the survival rate of human TSCC patients have not been clarified [15, 16]. At present, there is no TSCC cell line transfected with HPV16, which is indispensible for the further research. Considering that the TSCC cell line is the most common oral cancer and the site with the highest HPV infection rate in oral cancer (Table 1), it is necessary to establish this type of cell line for further research in the correlation between HPV and TSCC [17–19]. Therefore, we decided to establish and identify TSCC cell lines stably transfected with HPV16 E6 and E7 genes, in order to build an effective research model and observe the signaling pathways and pathogenic mechanisms of HPV16-related TSCC.

## 2. Materials and Methods

### 2.1. Information of Plasmid DNA including Fusion Gene E6E7 of HPV16

The ORF sequence of the fusion gene E6E7 for construction refers to the origin from GeneBank and then synthesized by GeneCopoeia in America. After picking and modifying, the final sequence application in the construction of ORF of rebuilding plasmid is ATGCACCAAAAGAGAACTGCAATGTTTCAGGACCCACAGGAGCGACCCAGAAAGTTACCACAGTTATGCACAGAGCTGCAAACAACTATACATGATATAATATTAGAATGTGTGTACTGCAAGCAACAGTTACTGCGACGTGAGGTATATGACTTTGCTTTTCGGGATTTATGCATAGTATATAGAGATGGGAATCCATATGCTGTATGTGATAAATGTTTAAAGTTTTATTCTAAAATTAGTGAGTATAGACATTATTGTTATAGTTTGTATGGAACAACATTAGAACAGCAATACAACAAACCGTTGTGTGATTTGTTAATTAGGTGTATTAACTGTCAAAAGCCACTGTGTCCTGAAGAAAAGCAAAGACATCTGGACAAAAAGCAAAGATTCCATAATATAAGGGGTCGGTGGACCGGTCGATGTATGTCTTGTTGCAGATCATCAAGAACACGTAGAGAAACCCAGCTGATGCATGGAGATACACCTACATTGCATGAATATATGTTAGATTTGCAACCAGAGACAACTGATCTCTACTGTTATGAGCAATTAAATGACAGCTCAGAGGAGGAGGATGAAATAGATGGTCCAGCTGGACAAGCAGAACCGGACAGAGCCCATTACAATATTGTAACCTTTTGTTGCAAGTGTGACTCTACGCTTCGGTTGTGCGTACAAAGCACACACGTAGACATTCGTACTTTGGAAGACCTGTTAATGGGCACACTAGGAATTGTGTGCCCCATCTGTTCTCAGAAACCATAG. The original GeneBank accession numbers referred are MN148319.1 and MK343347.1.

The plasmid vector with antibiotic resistant of Ampicillin, green fluorescent protein gene for fluorescence microscope, and stable selection maker of puromycin carrying about the ORF was then amplified using DH5*α* and extracted (Figure 1). At the same time, the empty vector plasmid was amplified and extracted by using the same method. The target plasmid was named pEGFP/HPV16 E6E7, and the empty vector plasmid was named pEGFP/no HPV16 E6E7, and both were stored in a -80°C refrigerator prepared for the transfection to oral squamous cell carcinoma cell lines.

The pEGFP/HPV16 E6E7 and the pEGFP/no HPV16 E6E7 were originally analyzed by DNA gel electrophoresis to explore the expression status of both of them (the figure was not shown here). In the end, the whole plasmid designed for this experiment was sent to check if the whole sequence was right and whether the condition of expression of the target plasmid was fine.

### 2.2. Transfection

Plasmids were transfected into tongue squamous cell carcinoma cells by liposome (lipo2000, Thermo Fisher Scientific, USA) transfection and then passed to a 96-well plate. The resistant cells were screened by puromycin.

### 2.3. Fluorescence Imaging after Transfection

After one day of passaging, SCC9 and SCC15 were, respectively, transfected with the pEGFP/HPV16 E6E7. Both of them were cultured in 1 mL culture medium, and after a period, the culture medium was changed. After a further culture for 48 h, all cells including SCC9 and SCC15, respectively, transfected with the pEGFP/HPV16 E6E7 were analyzed by both the dark field images and the bright field images under the fluorescence microscope.

### 2.4. Polymerase Chain Reaction (PCR) and Electrophoresis Analysis of Target Band Size

After transfection, the transfected cells were isolated with RNAiso reagent (Takara, Kyoto, Japan) to obtain the total corresponding RNA, and then the reverse transcriptional cDNA was obtained by PrimeScript RT reagent kit with gDNA Eraser (Takara, Kyoto, Japan), and then HPV16 forward primer 5′-ATGCACCAAAAGAGAACTGCAATG-3′ and HPV16 reverse primer 5′-CTATGGTTTTCTGAGAACAGATGGGGC-3′ were used, respectively (Table 2). The PCR were performed with Ex Taq (Takara, Kyoto, Japan). According to the instructions, after the corresponding reagents were PCR amplification, the reaction conditions were as follows: predenaturation at 94°C for 3 min, followed by 35 cycles at 94°C for 30 s and 65°C for 20 s, and extension at 72°C for 20 s and a final extension at 72°C for 5 min. The amplified product was obtained, and the size of the amplified product was analyzed by electrophoresis. The experiment was repeated for 3 times.

### 2.5. Cell Culture and Western Blot Analysis for E6/E7

The SCC9 and SCC15 were kindly provided by Dr. Wang of Guanghua Stomatologic College of Sun Yat-sen University. Cells were cultured in Ham's F12 nutrient medium/Dulbecco's modified Eagle's medium mixed with 10000 U/mL streptomycin (100x), 10 mg/mL penicillin (100x), and 10% fetal bovine serum.

Before the beginning of transfection, all passage cells should have been cultured for 12 h. After the transfection of pEGFP/HPV16 E6E7 and the pEGFP/no HPV16 E6E7 separately into SCC9 and SCC15, the puromycin was adopted to screening of cells with high expression of the puromycin resistance in order to pick out the cells with stable expression of pEGFP/HPV16 E6E7 and the pEGFP/no HPV16 E6E7.

After transfection, SCC9 and SCC15 transfected with the pEGFP/HPV16 E6E7,pEGFP/no HPV16 E6E7，and the no pEGFP/HPV16 E6E7 were washed by PBS three times and added to radioimmunoprecipitation assay (RIPA) lysis buffer (Thermo Fisher Scientific, Waltham, MA, USA) to obtain total protein. Then, the collected protein samples were separated by 12% SDS-poly-acrylamide gel electrophoresis (SDS-PAGE) and transferred onto polyvinylidene difluoride (PVDF) membrane (Millipore, Billerica, MA, USA). After being blocked with 5% nonfat milk powder at room temperature, the polyvinylidene difluoride membrane were incubated with primary antibodies against E6/E7 (monoclonal antibody of mouse anti-HPV E6/E7, Abcam) at 4°C overnight. Next, the membranes were washed with Tris-Buffered Saline Tween-20 (TBST) for 3 times, followed by incubation with anti-mouse Ig horseradish peroxidase linked secondary antibody (Proteintech, Chicago, IL, USA) at room temperature for 2 hours. The membranes were washed again with TBST for 3 times. Immunoreactive bands were detected by enhanced chemiluminescence (ECL) (Millipore, Billerica, MA, USA).

### 2.6. Cell Proliferation

The SCC9 and SCC15 were diluted into 5 × 10^4^/mL, and 100 *μ*L of the cell suspension was taken to passage in 96-well plates and was transfected with pEGFP/HPV16 E6E7 and the pEGFP/no HPV16 E6E7 12 h later. After being cultured for 6 h, 12 h, 18 h, and 24 h, all cells were detected by using CCK8 (Dojindo, Kumamoto, Japan).

### 2.7. State of Extensive Migration

The SCC9 and SCC15 were diluted into 10 × 6/mL, and 500 *μ*L of the cell suspension was taken to passage in 6 well plates and was transfected with pEGFP/HPV16 E6E7 and the pEGFP/no HPV16 E6E7 12 h later. A straight wound was caused by scraping the SCC9 and SCC15 with a 10 *μ*L pipette tip; the cells were washed three times with medium and then cultured in new complete medium. After being cultured for 0 h, 12 h, and 24 h, all cells were detected by a microscope.

### 2.8. RNA Extraction and Quantitative Real-Time PCR (qRT-PCR)

After transfection, the transfected cells were isolated with RNAiso reagent (Takara, Kyoto, Japan) to obtain the total corresponding RNA, and then the reverse transcriptional cDNA was obtained by PrimeScript RT reagent kit with gDNA Eraser (Takara, Kyoto, Japan). And then MMP2 forward primer 5′-CGTCTGTCCCAGGATGACATC-3′ and MMP2 reverse primer 5′-TGTCAGGAGAGGCCCCATAG-3′, MMP9 forward primer 5′-TGGGCAGATTCCAAACCTTT-3′ and MMP9 reverse primer 5′-TCTTCCGAGTAGTTTTGGATCCA-3′, and GAPDH forward primer 5′-GCTCTCTGCTCCTCCTGTTC-3′ and GAPDH reverse primer 5′-ACGACCAAATCCGTTGACTC-3′ (Table 2) were used, respectively. Real-time PCR was performed using SYBR Premix Ex Taq II (Takara, Kyoto, Japan) by Analytik Jena qTower 3g touch. According to the instructions, the reaction conditions were as follows: predenaturation at 95°Cfor 30 s, followed by 35 cycles at 95°C for 5 s, 55°C for 15 s, and 72°C for 30s. The data were collected and analyzed using the 2^-*ΔΔ*Ct^ method. The experiment was repeated for 3 times.

### 2.9. Cell Culture and Western Blot Analysis for MMP2/MMP9

The SCC9 and SCC15 were cultured in Ham's F12 nutrient medium/Dulbecco's modified Eagle's medium mixed with 100 U/mL streptomycin, 100 U/mL penicillin, and 10% fetal bovine serum.

Before the beginning of transfection, all passage cells should have been cultured for 12 h. After the transfection of pEGFP/HPV16 E6E7 and the pEGFP/no HPV16 E6E7 separately into SCC9 and SCC15, the puromycin was adopted to screening of cells with high expression of the puromycin resistance in order to pick out the cells with stable expression of pEGFP/HPV16 E6E7 and the pEGFP/no HPV16 E6E7.

After transfection, SCC9 and SCC15 transfected with the pEGFP/HPV16 E6E7 and the pEGFP/no HPV16 E6E7 were washed by PBS three times and added to radioimmunoprecipitation assay (RIPA) lysis buffer (Thermo Fisher Scientific, Waltham, MA, USA) to obtain total protein. Then, the collected protein samples were separated by 12% SDS-poly-acrylamide gel electrophoresis (SDS-PAGE) and transferred onto polyvinylidene difluoride (PVDF) membrane (Millipore, Billerica, MA, USA). After being blocked with 5% nonfat milk powder at room temperature, the polyvinylidene difluoride membrane were incubated with primary antibodies against MMP2/MMP9 (monoclonal antibody of mouse MMP2/MMP9, Abcam) at 4°C overnight. Next, the membranes were washed with Tris-Buffered Saline Tween-20 (TBST) for 3 times, followed by incubation with anti-mouse Ig horseradish peroxidase linked secondary antibody (Proteintech, Chicago, IL, USA) at room temperature for 2 hours. The membranes were washed again with TBST for 3 times. Immunoreactive bands were detected by enhanced chemiluminescence (ECL) (Millipore, Billerica, MA, USA).

### 2.10. Statistical Analysis

All results are expressed as the mean ± SD of triplicates in three independent experiments. Samples were analyzed by one-way analysis of variance (ANOVA) followed by the Newman–Keuls multiple range test (parametric). The acceptable level of significance was established at *p* < 0.05.

## 3. Results

### 3.1. Stability Detection

The lethal dose of SCC9 was 0.5 *μ*L/mL, and that of SCC15 was 3 *μ*L/mL. The selected epigenesis cells were further cultured for a normal passage. After a week of addition of puromycin, the cells all grew normally and the stability was verified.

### 3.2. Identification of Recombination Plasmid

The target sequence inserted into the plasmid vector which was designed for high expression of the fusion gene HPV16E6E7 was detected by the application of gene sequence analysis. Through observing the peak to valley profile of the target sequence, we can draw a conclusion that the expression of the target gene was exactly correct and could be stably expressing. The sequence analysis result was shown in the below peak-valley graph (Figure 2).

### 3.3. Identification of Transfection

To make sure the transfection efficiency was sufficient, all cells were taken photos by both the dark field images and the bright field images under the fluorescence microscope after appropriate transfection. Through the pictures taken in both the dark images and bright field, we can get the information of the transfection efficiencies of the two oral squamous cell carcinoma (OSCC) cell lines which were more than 80% (Figure 3).

### 3.4. Target Band Size of the Optimized Recombinant Fusion Gene Detection by Electrophoresis Analysis

SCC9 and SCC15 were, respectively, transfected with the synthetic gene pEGFP/HPV16 E6E7 and the pEGFP/no HPV16 E6E7. DNA sequencing assay revealed that the synthetic gene pEGFP/HPV16 E6E7 and the pEGFP/no HPV16 E6E7 were exactly the same as designed. As it was shown in Figure 4, the target band about 771 bp was exactly in the expected length (Figure 4). This suggests that the synthetic gene pEGFP/HPV16 E6E7 and the pEGFP/no HPV16 E6E7 had been constructed successfully.

### 3.5. Western Blotting Assay for Identify

As shown in Figure 5, Target Gene Prediction Software predicted that SCC9 and SCC15 transfected with the pEGFP/HPV16 E6E7,pEGFP/no HPV16 E6E7，and the no pEGFP/HPV16 E6E7 were, respectively, expressing correct proteins. The results showed that SCC9 and SCC15 transfected with the pEGFP/HPV16 E6E7 could stably express the target proteins and SCC9 and SCC15 transfected with the pEGFP/no HPV16 E6E7 express no target proteins.. The SCC9 and SCC15 transfected with no pEGFP/HPV16 E6E7 also express no target proteins. Till then, SCC9 and SCC15 transfected with the pEGFP/HPV16 E6E7,pEGFP/no HPV16 E6E7 and the no pEGFP/HPV16 E6E7 were expected to be expressing correct proteins which were finally steadily established.

### 3.6. Situation of Proliferation

CCK8 was adopted to evaluate the proliferation of SCC9 and SCC15 transfected with the pEGFP/HPV16 E6E7 and the pEGFP/no HPV16 E6E7. According to the results, it could be found that SCC9 transfected with the pEGFP/HPV16 E6E7 was growing faster than SCC9 transfected with the pEGFP/no HPV16 E6E7. Similarly, SCC15 transfected with the pEGFP/HPV16 E6E7 was growing faster than SCC9 transfected with the pEGFP/no HPV16 E6E7 (Figure 6).

### 3.7. Condition of Migration

As shown in Figure 7, SCC9 transfected with the pEGFP/HPV16 E6E7 migrated more quickly than the pEGFP/no HPV16 E6E7. Likewise, SCC15 transfected with the pEGFP/HPV16 E6E7 migrated more quickly than SCC9 transfected with the pEGFP/no HPV16 E6E7. But SCC9 transfected with the pEGFP/HPV16 E6E7 migrated much more quickly than SCC15 transfected with the pEGFP/HPV16 E6E7 (Figure 7).

### 3.8. Quantitative Real-Time PCR (qRT-PCR)

As expected, it was shown in Figure 7 that MMP2 and MMP9 were both expressed more in the SCC9 and SCC15 transfected with the pEGFP/HPV16 E6E7 than the cells transfected with the pEGFP/no HPV16 E6E7, which supports the migration discovery above (Figure 7).

### 3.9. Western Blotting Assay for Matrix Metalloproteinases

MMP2 and MMP9 were both expressed more in the SCC9 and SCC15 transfected with the pEGFP/HPV16 E6E7 than the cells transfected with the pEGFP/no HPV16 E6E7.

Target Gene Prediction Software showed that SCC9 and SCC15 transfected with the pEGFP/HPV16 E6E7 could express more matrix metalloproteinases including MMP2 and MMP9 than SCC9 and SCC15 transfected with the pEGFP/no HPV16 E6E7. Till then, SCC9 and SCC15 transfected with the pEGFP/HPV16 E6E7 and the pEGFP/no HPV16 E6E7 show more stability of migration than SCC9 and SCC15 transfected with the pEGFP/no HPV16 E6E7 (Figure 8).

## 4. Discussion

It was found that people with more sex partners, with increasing intensity (per month), with longer duration (in years), and with more cultivative joint-years all could be more possible to be exposed to HPV16-positive HOSCC [20]. And studies confirming that there was high frequency detection of HPV DNA in HOSCC which were more numerous by Southern blot hybridization, polymerase chain reaction, and in situ hybridization and through collection of clinical evidence. What is more, it was proved that there was a stronger relation between HPV oral infection and couples who had ever have oral sex or open-mouthed kissing than others who just had vaginal sex [21].

As for the treatments of OSCC, surgery, as a frequent and destructive treatment, was still the basic optional therapy for almost all of the cancers. It was reported that cold knife, electrosurgery, laser therapy, and large loop excision of transformation zone were suitable for genital mucosa while cold knife, quantic molecular resonance scalpel, electro-surgery, and laser therapy were specifically adopted on the therapy of oral mucosa. Ablative destructive therapy including cryotherapy, monobromoacetic acid, bromochloroacetic acid, trichloroacetic acid, aldehydes, salicylic acid, and photodynamic therapy was advisable for the treatment of genital mucosa. Antiproliferant, cytotoxic, and antiviral agents are composed of podophyllin, podophyllotoxin, 5-FU, and cidofovir. In addition to immunomodulator agents including imiquimod, IFN*α*, and IFN*β* and novel therapies including ribozymes, siRNA, and antisense oligonucleotides, molecular targeted therapy was also available for the treatment of genital mucosa.

Subsequently, HPV-related carcinoma was still a big deal for exploration particularly on clinical therapeutic methods which could not have breakthrough in the last decades. Among the studies on searching target point for the development of new drugs, E6 and E7 remain the two major essential oncogenes for the development and maintaining malignancy on HPV-associated human cancers, which were attractive functional inhibition and specific therapeutic target [22, 23]. In decades, there were numbers of therapeutic methods targeting either E6 or E7 which have been deeply explored by retrospective analysis and hypothesis tests through both experimental and clinical study hypotheses. Nowadays, it was gradually proved that treatment modalities targeting both E6 and E7 had better curative effect than targeting either alone [24, 25]. Therefore, molecular E6/E7 was the most accurate curation with high efficacy and low toxicity and had significant curative effect target among the novel therapies presented above, which was deserved to be further studied [26].

But there is no oral squamous cell line transfected with HPV currently, in which it is not conducive to study the connection between HPV and oral squamous cell cancer and develop the novel treatment of HPV-related OSCC. So it was particularly necessary for us to establish a stable oral squamous cell line transfected with HPV for a further study of HPV-related OSCC. As the TSCC cell line is the most common oral cancer and the site with the highest HPV infection rate in oral cancer, it is necessary to establish this type of cell line. But TSCC cell lines transfected with HPV16 E6E7 were inexistent in the decades, which was really a developmental limitation for a further study on the pathological mechanism, preventive measures, and treatment protocols of oral cancers, with the finding that E6 and E7 showed increasing expression as the HPV16 infection increased [27]. In this study, we transfer the pEGFP/HPV16 E6E7 and the pEGFP/no HPV16 E6E7 into TSCC cells separately, to establish a stable HPV-transferred TSCC cell line and further confirm the possible role of E6 and E7. The analysis results showed that the synthetic gene the pEGFP/HPV16 E6E7 and the pEGFP/no HPV16 E6E7 had been constructed successfully and they, respectively, transfected into SCC9 or SCC15 efficiently.

To further evaluate the effects of E6 and E7 on HPV-related OSCC, it was found that SCC transfected with the pEGFP/HPV16 E6E7 was growing and migrating faster than the SCC transfected with pEGFP/no HPV16 E6E7, which means E6/E7 was able to stimulate the growth and migration of squamous cell carcinoma cells. Furthermore, the qRT-PCR analysis showed that matrix metalloproteinases including MMP2 and MMP9 were both expressed more in the TSCC transfected with the pEGFP/HPV16 E6E7 than the pEGFP/no HPV16 E6E7 group. And the E6/E7 group promoted the migration of TSCC. And these findings illustrated that HPV16 E6/E7 gene silencing could avoid ability enhancement of the proliferation and migration of TSCC cells, which is a conclusive evidence about the promising clinical effect of E6/E7-targeted molecules.

## 5. Conclusion

In conclusion, TSCC cell lines infected with HPV16 E6E7 showed significantly higher ability of proliferation and migration than those not infected with HPV16 E6E7. And this reflects the possibility that the E6/E7 inhibitors might have the effects on suppressing carcinoma clinically. But its complete signal pathway and mechanisms remain to be discovered clearly if needed to further apply these findings to clinical practice.

## Figures and Tables

**Figure 1:** Vector information for recombinant plasmid pEGFP/HPV16 E6E7.

**Figure 2:** Stability analysis of ORF sequence information for recombinant plasmid pEGFP/HPV16 E6E7.

**Figure 3:** Fluorescence imaging after transfection in both the dark field images and the bright field. SCC9 transfected with the pEGFP/HPV16 E6E7 under the dark field images (a). SCC15 transfected with the pEGFP/HPV16 E6E7 under the dark field images (b). SCC9 transfected with the pEGFP/HPV16 E6E7 under the bright field images (c). SCC15 transfected with the pEGFP/HPV16 E6E7 under the bright field (d).

**Figure 4:** Analysis of the expression plasmid pEGFP/HPV16 E6E7 in SCC9 and SCC15. SCC9 transfected with the pEGFP/no HPV16 E6E7 (a). SCC9 transfected with the pEGFP/HPV16 E6E7 (b). SCC15 transfected with the pEGFP/no HPV16 E6E7 (c). SCC15 transfected with the pEGFP/HPV16 E6E7 (d).

**Figure 5:** Western blot detection of the expression of recombinant plasmid-no pEGFP/HPV16 E6E7, pEGFP/no HPV16 E6E7, and pEGFP/HPV16 E6E7 in SCC9 and SCC15.

**Figure 6:** Statistical analysis of the proliferative ability of SCC9 and SCC15 each transfected with the pEGFP/HPV16 E6E7 and the pEGFP/no HPV16 E6E7 (^∗^*p* < 0.05).

**Figure 7:** State of extensive migration. Imaging of migration situation of SCC9 and SCC15 transfected with the pEGFR/HPV16 E6E7 and the pEGFR/no HPV16 E6E7 (a). Statistical analysis of the migration capability of SCC9 and SCC15 transfected with the pEGFR/HPV16 E6E7 and the pEGFR/no HPV16 E6E7 (^∗^*p* < 0.05) (b). The relative expression of mRNA levels in SCC9 transfected with the pEGFP/no HPV16 E6E7 and SCC9 transfected with the pEGFP/HPV16 E6E7 and SCC15 transfected with the pEGFP/no HPV16 E6E7 and SCC15 transfected with the pEGFP/HPV16 E6E7 (^∗^*p* < 0.05) (c).

**Figure 8:** Western blot detection of the expression of MMP2 and MMP9 in SCC9 and SCC15 transfected with recombinant plasmid pEGFP/no HPV16 E6E7 and pEGFP/HPV16 E6E7 (a). The relative expression of protein-MMP2 and MMP9 in SCC9 transfected with the pEGFP/no HPV16 E6E7 and SCC9 transfected with the pEGFP/HPV16 E6E7 and SCC15 transfected with the pEGFP/no HPV16 E6E7 and SCC15 transfected with the pEGFP/HPV16 E6E7 (^∗^*p* < 0.05) (b).

**Table 1:** Characteristic data of the HPV virus detection in oral cancer.

Authors	Year	Country	Detection method	Case	HPV+		Male (HPV+)		HPV type (%)		HPV + tongue no./total tongue no.(%)
					*N*	%	*N*	%	16	18	
Balaram et al.	1995	India	PCR	91	67	74%	37	55%	38%	43%	82%
Jenice et al.	1998	India	PCR & Southern blot	100	15	15%	9	60%	100%	0	43%
Pillai et al.	1999	India	In situ hybridization & immunocytochemistry	61	39	64%					
Nagpal et al.	2002	India	PCR	110	37	34%	15	60%	23%	15%	33%
Jayasooriya et al.	2003	Sri Lanka	PCR	102	38	37%	28	74%	47%	7%	50%
Koppikar et al.	1999-2003	India	PCR	102	32	31%	25	37%	6%	6%	
Mishra et al.	2006	India	PCR	66	18	27%	57	86%	18%	0	67%
Castillo et al.	1996-2002	Pakistan	PCR & in situ hybridization	48	27	56%			100%	0	
Kulkarni et al.	2009-2010	India	PCR	34	24	71%			42%	22%	
Elango et al.	2004-2007	India	PCR	60	29	48%	22	76%			48%
Bahl et al.	2010-2011	India	PCR & in situ hybridization	105	24	23%	22	92%	79%	13%	40%
Nemes et al.	2006	Hungary	PCR	79	33	42%	30	91%	100%	0	
Syrjanen et al.	1962-1978	Finland	In situ hybridization	51	6	12%	2	33%	33%	50%	64%
Chang et al.	1990	Finland	PCR & in situ hybridization	40	12	30%			82%	9%	
Shindoh et al.	1988-1991	Japan	PCR	77	24	31%	17	71%	100%	0	
Cruz et al.	1996	Netherlands	PCR	35	19	54%	12	80%	79%	0	36%
Mao et al.	1996	USA	PCR	64	20	31%	15	75%	75%	20%	61%
Wen et al.	1997	Japan	PCR	45	14	30%			20%	24%	63%
Koh et al.	1989-1996	Korea	PCR	42	22	52%			68%	27%	
Schwartz et al.	1990-1995	USA	PCR	248	64	21%			95%	5%	
Aggelopoul-ou et al.	1999	Greece	PCR	81	40	50%			13%	55%	
Tsuhako et al.	1993-1996	Japan	PCR	83	48	57%			46%	38%	44%
Premoli-De-Percoco et al.	2001	Venezuela	PCR	50	30	60%			73%	17%	50%
Schwartz et al.	1988-1995	USA	PCR	254	62	24%	26	65%	16%		
Nsgpal et al.	1999-2002	India	PCR	110	37	34%	17	55%	23%	15%	33%
Chang et al.	1988-2002	China	PCR	103	51	50%	14	27%	57%	53%	
Ritchie et al.	1994-1997	USA	PCR	141	29	21%	8	28%	83%	3%	60%
Sugiyama et al.	1981-2000	Japan	PCR	86	30	35%	16	53%	100%	0	36%
Dahlgren et al.	1970-2002	Sweden	PCR	110	12	11%	10	83%	75%		
Chang et al.	1994-2011	China	PCR & dot blot hybridization & in situ hybridization	610	354	58%			47%		
Smith et al.	1994-1997	USA	PCR	193	38	20%	28	74%	87%		
Zhang et al.	1997-1999	China	PCR	73	54	74%	39	72%	67%	20%	80%
El-Mofty et al.	2006	USA	PCR; immunohistochemistry	20	12	60%			83%		
Nemes et al.	1996-2001	Hungary	PCR	79	33	42%	30	91%	82%		65%
Koyama et al.	2007	Japan	In situ hybridization & PCR	20	20	100%	11	55%	20%	45%	100%
Sugiyama et al.	1992-1999	Japan	PCR	66	24	36%	13	54%	100%	0	67%
Kuo et al.	1997-2005	China	Immunohistochemical & in situ hybridization & PCR	92	69	75%	56	81%	84%	3%	
Saini et al.	2011	Malaysia	PCR	105	54	52%	24	44%	74%		55%
Ma et al.	1998	China	PCR, Southern blot hybridization & immunohistochemical staining	102	60	59%			50%	37%	
Shima et al.	1991-1996	Japan	PCR	46	34	74%			20%	54%	
Angela et al.	1987-2006	Australia	PCR	411	185	46%	146	79%	95%		
Bhawal et al.	2008	Japan	PCR	29	11	38%	20	69%	100%	0	
Chen et al.	2012-2015	China	PCR	178	25	14%			24%	76%	
Anil et al.	1973-2004	USA	PCR	45769	17625	39%	12794	73%			
Mellin et al.	1984-1996	Sweden	PCR	60	26	43%	15	58%	100%	0	
Gan et al.	2009-2013	China	PCR	200	55	28%			71%	27%	

**Table 2:** Specific primers used in the present study.

Name	Forward (5′-3′)	Reverse (5′-3′)
HPV16	ATGCACCAAAAGAGAACTGCAATG	CTATGGTTTTCTGAGAACAGATGGGGC
MMP2	CGTCTGTCCCAGGATGACATC	TGTCAGGAGAGGCCCCATAG
MMP9	TGGGCAGATTCCAAACCTTT	TCTTCCGAGTAGTTTTGGATCCA
GAPDH	GCTCTCTGCTCCTCCTGTTC	ACGACCAAATCCGTTGACTC

## Data Availability

All date generated during this experiment are included in the article above.
